# Effect of Dihydroquercetin on Energy Metabolism in LPS-Induced Inflammatory Mice

This article has been retracted.

**DOI:** 10.1155/2022/6491771

**Published:** 2022-07-04

**Authors:** Xiaoying Yu, Saddam Hussein, Lijia Li, Qingyu Liu, Zhibin Ban, Hailong Jiang

**Affiliations:** ^1^Department of Animal Science and Technology, Jilin Agricultural University, Jilin Province, Changchun, China 130118; ^2^Jilin Academy of Agricultural Sciences, No. 1363 Shengtai Street, Changchun City, Jilin Province, China 1300119

## Abstract

This study investigated the effects and alterations of dihydroquercetin on the growth performance, nutriment metabolism, antioxidant and immune function, and energy substrate utilization in lipopolysaccharide-challenged mice. A total of 0, 50, and 200 mg/kg of dihydroquercetin were intragastrically administered once a day for 21 days. After the pretreatment with dihydroquercetin, each group was subjected to a lipopolysaccharide challenge (except for the control group). After lipopolysaccharide injection, food intake, body weight, metabolic indexes of blood and liver nutrients, blood inflammatory factors, and liver oxidative stress indexes were measured at 6, 12, 24, and 48 h, respectively. Indirect calorimetry analysis was performed by respiratory gas analysis for 48 h to calculate the energy substrate metabolism of carbohydrate, fat, and protein. Urinary nitrogen excretion was measured to evaluate the urinary protein metabolism to calculate the substrate utilization. The results showed that dihydroquercetin pretreatment can significantly increase the weight gain and average food intake and decrease the mortality rate in lipopolysaccharide-induced inflammation mice. Furthermore, dihydroquercetin pretreatment can alleviate the negative effects of lipopolysaccharides by increasing levels of superoxide dismutase and glutathione peroxidase and by decreasing the malondialdehyde and serum inflammatory cytokines (interleukin-1*β*, nuclear factor *κ*B, and interleukin-6). Dihydroquercetin pretreatment also can relieve nutrient metabolic disorder by increasing blood glucose, serum total protein, and liver glycogen levels and reducing serum and liver triglycerides, serum cholesterol, serum lactate dehydrogenase, and serum urea nitrogen levels. Meanwhile, it increases the relative utilization of carbohydrate, reducing relative utilization of protein and lipid, alleviating the change in energy metabolism pattern from glucose-predominant to lipid-predominant caused by lipopolysaccharide stimulation. In addition, the degree of metabolic pattern transformation depends on the dose of dihydroquercetin supplement. Finally, according to principal component analysis, we found that the inflammation was strongest in the mice at 24 h and was subsequently relieved in the LPS-stimulated group, whereas in the dihydroquercetin-pretreated group, the inflammation was initially relieved. To summarize, dihydroquercetin pretreatment can improve energy metabolism disorder and attenuate the negative effects of lipopolysaccharide challenge in mice from the initial stage of inflammation.

## 1. Introduction

The inflammatory state is associated with metabolic disorders of nutrients in the body [1]. The conversion of bioenergy materials closely links metabolism with inflammation and immunity to protect cells and organisms and promote the restoration of balance [2]. The early initial stage of acute inflammation is anabolic, which mainly maintains a high energy demand by increasing glycolysis and reducing mitochondrial glucose oxidation for energy [3]. Even in the presence of oxygen, metabolic reprogramming with glycolytic metabolic energy supply is the priority. This is known as the Warburg effect [4]. The adaptation (recovery) stage is dominated by catabolism, which mainly needs fatty acid oxidation to obtain energy [5] and depends on fatty acid oxidation to heal and restore the balance of the body [6, 7]. This reprogramming of the glycolytic and fatty acid oxidation metabolic pathways provides the required energy for both the early initiation proinflammatory phase and the later adaptive phase in acute inflammation. However, in clinical research, it is difficult to timely predict the degree of changes in and types of energy substrate metabolism in patients under a persistent inflammation condition. Therefore, it is hard to understand the clinical course of the disease in time and to provide adequate treatment and administration plans for patients.

Indirect calorimetry (IC) is a noninvasive method for determining energy needs and the rate of energy substrate consumption from the consumption and production gas. This analysis based on the laws of energy conservation and of definite proportion in chemical reactions [8]. Animals' energy metabolism is affected by many factors, such as disease, temperature, hunger, and exercise. On the contrary, monitoring the consumption of carbohydrates, lipids, and proteins as energy substrates in animals can directly reflect the health status of organisms [9]. Under normal physiological conditions, an organism's energy intake and consumption maintain a stable balance, which is a prerequisite for ensuring health. In the acute phase, the balance between catabolism and anabolism is broken, which changes the metabolic law of the three nutrients; this is directly reflected in changes in CO_2_ exhalation, O_2_ consumption, and nitrogen excretion. Given the noninvasive nature and immediacy of data acquisition, this method has been validated as an objective and convenient adjunct to metabolic assays, is flexible enough to be combined with other methods, and has been used to investigate mechanisms such as nutrition [10–12], energetics of physical exercise [13], obesity [14, 15], or other metabolic diseases [16, 17]. It is also widely used in modern clinical medicine (such as in acute illness, intensive care [18], and parenteral nutrition [19, 20]). However, research combined with the study of drug treatment or prevention effects is still relatively rare.

Dihydroquercetin (DHQ) (3,3′,4′,5,7-pentahydroxyflavanone) belongs to the flavone subclass of flavonoids, with a yellow powder or colorless needle crystal appearance and no special smell, as shown in Figure 1. It is a well-soluble in organic solvent such as DMSO but less soluble in water [21]. It was first extracted from the heartwood of Douglas fir bark [22] and is also be found widely in Japanese Larch [23], Siberian larch (Larix sibirica), onion [24], milk thistle [25], and rosette [26]. In recent years, studies have reported that DHQ has excellent antioxidant, anti-inflammatory, antibacterial, and anticancer properties, like other flavonoids. At present, it is also widely used as a food additive and in health supplement commercial products such as silymarin (Legalon) ™) and Pycnogenol ®. However, as we acknowledge, it has been rarely reported that DHQ, as an immune booster, has an impact on animal protection and regulation of energy metabolism under inflammatory responses. Therefore, the purpose of our study was to examine the protective effect of DHQ by detecting the dynamic changes and effects of DHQ on growth, antioxidation, immune response, and energy metabolism in mice under LPS attack.

## 2. Materials and Methods

The experiment was carried out in Jilin Academy of Agricultural Sciences, Changchun, China. All the experimental animals used were used in accordance with the NIH Guide for the Care and Use of Laboratory Animals. This study was carried out in strict accordance with the recommendations in the Guide for the Care and Use of Laboratory Animals of the National Institutes of Health.

### 2.1. Animals and Treatment

Male 6-week-old BALB/c mice (*n* = 92) were purchased from the Changchun Yisi Laboratory Animal Technology Co. Ltd. (Changchun, China). Mice were given ad libitum access to water and food and were housed at a temperature of 22 ± 2°C and relative humidity of 60% ± 10% with 12 h light/12 h dark for a total rearing period of 23 days. After a 5-day acclimation period, mice were divided into four different treatments groups (*n* = 23 mice per group) according to the principle of weight average, and 5–6 mice were housed in a feeding cage with bedding material. The four groups were the control group (C), LPS model group (C+), low-dose treatment group (DHQ-L, 50 mg/kg BW of DHQ), and high-dose treatment group (DHQ-H, 200 mg/kg BW of DHQ). DHQ (Sengong, JILIN, Changchun, China) was dissolved in sodium carboxymethyl cellulose (CMC-NA) and administered to mice by oral gavage for the two DHQ treatment groups, whereas the groups C and C+ were gavaged with an equal volume of CMC-NA and continuously fed for 21 d at a fixed time.

On day 21, groups C+, DHQ-L, and DHQ-H were injected with an equal volume of LPS (Escherichia coli O55, B5 L-2880; Sigma-Aldrich, USA) at a dose of 2.5 mg/kg BW/mouse, and group C was injected with an equal volume of saline to establish the inflammatory model. Euthanasia and laparotomy were performed at 6 h, 12 h, 24 h, and 48 h after LPS injection.

All protocols of animal care and experiments were performed in accordance with the Animal Research: Reporting of In Vivo Experiments (ARRIVE) guidelines [27].

### 2.2. Animal Samples and Data Collection

Next, 0, 24, and 48 h after LPS/normal saline injections, the number of deaths, the average daily gain (ADG), and average daily feed intake (FI) of the mice were recorded in each group.

Blood sample collection was performed at each time point of 6 h, 12 h, 24 h, and 48 h after LPS/saline injection (4–5 mice were randomly collected from each group in the first 3 time points and 6–8 mice were collected from each group at 48 h) and collected in polypropylene tubes. Serum was obtained by centrifugation at 3000 rpm/min for 15 min under 4°C and then stored at −20°C until analysis. After LPS/saline injection, urine samples were collected every 6 h in metabolic cages and a mixture of samples every 24 h was stored at −20°C after centrifugation. Liver samples were collected after collecting blood at each time point of 6 h, 12 h, 24 h, and 48 h. The residual blood was washed away in ice-cold saline, the fascia and fat were shaved, blotted with filter paper and weighed, and then stored frozen at −80°C in aliquots. Indirect calorimetry data collection began on the 19th day of environmental acclimatization. Six mice were selected per treatment group, and every two were housed in one respiratory thermometry chamber. The formal test started after LPS/saline injection and was monitored continuously for 48 h, during which the exhaled CO_2_ and consumed O_2_ data for each chamber were recorded by a computer every 18 min.

### 2.3. Detection Method and Calculation Formula

The content of blood glucose (Glu), triglyceride (TC), total cholesterol (TG), serum total protein (TP), serum urea nitrogen (BUN), and lactate dehydrogenase (LDH) in serum were evaluated by an automatic blood biochemical analyzer (Hitachi 7060). Liver glycogen and liver triglyceride contents were assessed using commercial kits (Nanjing Jiancheng Bioengineering Institute, Nanjing, China) according to manufacturer's instructions. Urine was diluted to 50 mL with distilled water, and urea nitrogen content was determined using a commercial kit based on the diacetyl monoxime colorimetry method (Nanjing Jiancheng Bioengineering Institute, Nanjing, China). Urine nitrogen emission (mg/d) = urea concentration (mg/L) × 0.05 × 28 g/mol ÷ 60 g/mol. Note: 28 g/mol is the molecular weight of N_2_ and 60 g/mol is the molecular weight of urea.

The serum levels of TNF-*α*, IL-6, and IL-1*β* were measured using enzyme-linked immunosorbent assay (ELISA) with commercially available kits (Enzyme-linked Biotechnology Co. Ltd., Shanghai, China), following the manufacturer's instructions.

The open-circuit respiration chambers in parallel were used to measure oxygen consumption and carbon dioxide exhalation, which has been previously described by Liu et al. [28]. A controlled-temperature device was installed inside the chamber to maintain a constant operating temperature and humidity, and then, gas exchange measurements for each chamber were recorded every 3 min on a computer, and mean values for every 6 h period were used for the analysis. The O_2_ was measured with a zirconium oxide sensor (Model 65-4-20; Advanced Micro Instruments, Huntington Beach, CA, USA), and a nondispersive infrared sensor (AGM 10; sensors Europe GmbH, Erkrath, Germany) was used for CO_2_ measurement. The indirect calorimeter consists of a sealed transparent glass chamber with a variable flow through the chamber, connected to a nondispersive infrared sensor (AGM 10; sensors Europe GmbH, Erkrath, Germany) to measure CO_2_ exhalation and a zirconium oxide sensor (Model 65-4-20; Advanced Micro Instruments, Huntington Beach, CA, USA) to measure O_2_ consumption.

The respiratory quotient (RQ), total energy expenditure (TEE), carbohydrate oxidation (CHO), fat oxidation (FAO) and protein oxidation (PRO), energy provided by carbohydrate oxidation (OXCHO), energy provided by fat oxidation (OXF), and energy provided by protein oxidation (OXP) were calculated according to the following formula:

(1) $$\begin{array}{c} \text{RQ}=\frac{{\text{VCO}}_{2}\left(\text{L}/\min\right)}{{\text{VO}}_{2}\left(\text{L}/\min\right)}, \end{array}$$

TEE (kcal/min) = 3.816 × VO2 (L/min) + 1.231 × VCO2 (L/min)–1.889 × N (Lusk′s formula), [29]

CHO (mg) = 4.55 × VCO2 (L/min) − 3.21 × VO2 (L/min) − 2.87 × N (Frayn′s formula), [30]

FAO (mg) = 1.67 × (VO2–VCO2) − 1.92 × N (Frayn′s formula), [30]

PRO (mg) = N (mg/h) × 6.25,

OXCHO (kcal/min) = CHO × 4.2,

OXF (kcal/min) = FAO × 9.5,

OXP (kcal/min) = PRO × 4.4,

Proportion of carbohydrate oxidation energy supply = CHO × (4.2/TEE), 

Proportion of fat oxidation energy supply = FAO × (9.5/TEE), 

Proportion of protein oxidation energy supply = PRO × (4.4/TEE).

### 2.4. Statistical Analysis

All data in this study are presented as means plus standard deviation. Data were analyzed using SPSS 21.0 software (IBM, Chicago, IL, USA). Correlation analysis was performed with R and processed for data visualization. Spearman's method was used for correlation analysis. Principal component analysis was performed with R, and data processing and visualization were performed. The data were analyzed using a one- or two-way analysis of variance (ANOVA) with Tukey's post hoc tests to determine the significant differences between group means. The level of significance was considered as *p* < 0.05.

## 3. Result

### 3.1. Growth

In our study, a mouse inflammatory model was established by the intraperitoneal injection of LPS to explore the protective effect of DHQ pretreatment against inflammatory challenge. In the survival analysis, mice in groups C+ and DHQ-L began to perish 6 h after LPS injection, and the survival rate of these mice at 48 h was 91.3% and 95.6%, respectively. In contrast, the survived rates of groups C and DHQ-H were 100% within 48 h after LPS injection, as shown in Figure 2(a). The results of the average daily gain (ADG) and daily feed intake (FI) of mice are also shown in the figure, as shown in Figures 2(b) and 2(c). Compared to group C, in the LPS treatment groups, the ADG and FI were decreased significantly (*p* < 0.01) within 2 days, whereas compared with the C+ group, the ADG of the DHQ-H group was significantly increased (*p* < 0.05) within 2 days, and the FI of the DHQ-H group and the ADG of the DHQ-L group were significantly increased (*p* < 0.05) on the second day.

### 3.2. Metabolism of Nutrients in Serum and Liver

In contrast to those of the C group, the GLU in LPS-treated mice increased briefly and then decreased significantly at 12 h, 24 h, and 48 h (*p* < 0.05 or *p* < 0.01), as shown in Figure 3(a). However, in contrast to the C+ group, serum GLU in the DHQ pretreatment group increased significantly (*p* < 0.01) at 24 h and 48 h in a dose-dependent manner. Compared with group C, the contents of serum LDH, TC, TG, and BUN, as shown in Figures 3(b)–3(e), in the LPS-stimulated groups increased significantly (*p* < 0.05 or *p* < 0.01) within 48 h. Furthermore, compared with those of the C+ group, sera LDH, TC, TG, and BUN in the DHQ pretreatment group decreased in a dose-dependent manner at four time points, among which the DHQ-H group had statistical significance (*p* < 0.05 or *p* < 0.01). Compared with group C, serum TP in group C+ and DHQ-L increased significantly (*p* < 0.05 or *p* < 0.01), as shown in Figure 3(f), while that in group DHQ-H decreased significantly (*p* < 0.05) 12 h after LPS injection. At 24 h and 48 h, compared with group C, the serum TP in the other LPS-challenged groups decreased significantly (*p* < 0.01). However, in contrast to the C+ group, the serum TP level significantly increased in the DHQ-H group (*p* < 0.01). The content of liver glycogen is shown in Figure 3(g). Compared with group C, the hepatic glycogen content in each group after LPS stimulation was significantly decreased (*p* < 0.01). In contrast to the C+ group, liver glycogen content was significantly increased in the DHQ-H group (*p* < 0.05). Hepatic TG content, as shown in Figure 3(h), significantly increased in each group after LPS stimulation (*p* < 0.01). However, in contrast to the C+ group, levels in the DHQ-L group and the DHQ-H group were significantly decreased within 2 days (*p* < 0.05).

### 3.3. Antioxidant Index in Liver

As shown in Figure 4, the level of liver MDA significantly increased (*p* < 0.01) and the levels of liver SOD and GSH-Px significantly decreased (*p* < 0.01) in the LPS-stimulated group compared with those of the group C at four time points. Compared with group C+, the content of MDA in the DHQ-L group decreased significantly at 6 h, 12 h, and 24 h (*p* < 0.05 or *p* < 0.01), while in the DHQ-H group, it decreased significantly at 6 h, 12 h, 24 h, and 48 h (*p* < 0.05 or *p* < 0.01), as shown in Figure 4(a). The content of SOD in the DHQ-L group increased significantly at 12 h, 24 h, and 48 h (*p* < 0.05 or *p* < 0.01) and that in the DHQ-H group increased significantly at 6 h, 12 h, 24 h, and 48 h (*p* < 0.05 or *p* < 0.01), as shown in Figure 4(b). The content of GSH-Px in the DHQ-H group increased significantly at 6 h, 12 h, 24 h, and 48 h (*p* < 0.05), as shown in Figure 4(c).

### 3.4. Serum Inflammatory Cytokines

As shown in Figure 5, groups receiving LPS stimulation had significantly increased TNF-*α*, IL-1*β*, and IL-6 levels in their serum compared with the C group (*p* < 0.01) within 48 h. Compared with the C+ group, serum TNF-*α*, IL-1*β*, and IL-6 level decreased significantly in the DHQ-H group at four time points (*p* < 0.01 or *p* < 0.05). Moreover, in the DHQ-L group, serum IL-1*β* level decreased significantly at 6 h and 48 h (*p* < 0.01 or *p* < 0.05), and serum IL-6 decreased significantly at 6 h, 24 h, and 48 h (*p* < 0.01). In terms of time, after LPS injection, the level of inflammatory cytokines first increased and then decreased. At 12 h, the levels of TNF-*α*, IL-1*β*, and IL-6 in the serum were the highest and then began to decrease from 24 h.

### 3.5. Indirect Calorimetry Analysis

The results for O_2_, CO_2_, RQ, and TEE after LPS challenge are shown in Figure 6. In group C, mice displayed a basal circadian rhythm in which O_2_, CO_2_, RQ, and TEE were elevated during the dark phase (12–24 h/36–48 h) and decreased during the light phase (0–12 h/24–36 h). In contrast to group C, following LPS stimulation, the O_2_, CO_2_, RQ, and TEE significantly decreased (*p* < 0.01). The overall levels of each indicator first decreased, reached a nadir at 18–24 h, and then increased slowly, meaning the original circadian rhythm was broken. However, DHQ pretreatment could increase O_2_, CO_2_, RQ, and TEE compared to the C+ group in a dose-dependent manner at 6 h, 12 h, 24 h, and 48 h.

Subsequently, the substrate utilization values of carbohydrate, fat, and protein and their proportion of total energy consumption were calculated according to the formula, as shown in Figure 7. In contrast to group C, OXCHO and OXCHO/TEE significantly decreased (*p* < 0.01), and OXF, OXF/TEE, OXP, and OXP/TEE significantly increased (*p* < 0.01) in the LPS-stimulated groups at 6 h, 12 h, 24 h, and 48 h. Compared with the C+ group, OXCHO, OXCHO/TEE, and OXF increased in a dose-dependent manner, while OXF/TEE OXP, and OXP/TEE decreased in a dose-dependent manner in the DHQ pretreatment groups. Compared with the C+ group, the values of OXP (day1 and day2) and OXP/TEE (at 6 h, 12 h, 24 h, and 48 h) were significantly decreased in the DHQ-L group (*p* < 0.01 or *p* < 0.05). The values of OXCHO (6 h, 12 h, 24 h, and 48 h), OXCHO/TEE (24 h and 48 h), and OXF (6 h and 12 h) were significantly increased (*p* < 0.01 or *p* < 0.05), and OXF/TEE (12 h, 24 h, and 48 h), OXP (day1 and day2), and OXP/TEE (6 h, 12 h, 24 h and 48 h) were significantly reduced (*p* < 0.01 or *p* < 0.05) in the DHQ-H group. Notably, after LPS injection, OXCHO and OXCHO/TEE decreased first and then increased, reaching their lowest point at 24 h. OXF/TEE and OXP showed a trend of first increasing and reaching the peak at 24 h, and then decreasing, while OXF decreased continuously with time.

### 3.6. Principal Component Analysis (PCA)

In a previous study, we showed that the administration of LPS to mice and pretreatment with DHQ could cause changes in cytokine indicators, antioxidant indicators, and growth performance indicators and could also affect energy metabolism. To explore the association between several clinical and energy metabolism indicators, we performed correlation analysis between 22 indicators in the above four broad categories, and the data were visualized and processed as shown in Figure 8. There was a significant positive correlation (*p* < 0.01) between TG, TC, bun, MDA, IL-1*β*, IL-6, TNF-*α*, and OXP/TEE, OXF, OXP, and OXF/TEE, whereas a significant negative correlation was observed between OXCHO, OXCHO/TEE, O_2_, and CO_2_ (*p* < 0.01). GSH-Px, SOD, ADG, and FI showed a significant negative correlation (*p* < 0.01) with OXP/TEE, OXF, OXP, and OXF/TEE, and a significant positive relationship (*p* < 0.01) with OXCHO, OXCHO/TEE, O_2_, and CO_2_.

Subsequently, principal component analysis (PCA) was performed on the results of 22 indicators in the four treatment groups at four time points, and the results are shown in Figure 9. The contributions of PC1 and PC2 can explain 74.2% and 11.9% of the cumulative variables in the data, respectively, and could well represent most characteristic information of the original data. The contributions of various indexes to the principal components are shown in Figure 9(a). The larger the COS_2_ value, the greater the contribution. There was also an obvious classification among various indicators; the positively correlated variables were relatively close to each other, and the negatively correlated variables were distributed toward both ends through the origin. When the indices of daily weight gain, feed intake, O_2_, C O_2_, OXCHO, OXCHO/TEE, GLU, SOD, and GSH-Px were compared with the indices of TG, TC, LDH, BUN, TNF-*α*, IL-1*β*, IL-6, OXF/TEE, OXP, OXP/TEE, OXF, and MDA presented a clear negative relationship. As shown in Figure 9(b), different colors represent different treatment groups, different shapes represent different time points, and a closer distance between two points indicates less dissimilarity.

The points representing LPS stimulation in the different treatment groups were far away from group C, illustrating that LPS has an obvious effect on mice. However, there was also a clear separation between the groups given LPS stimulation, in which the DHQ-H group was closer to the C group than to the other groups, which indicated that DHQ pretreatment and dosage also had an effect on the mice. Combined with the Figure 9(a), the closer a point is to the left of the coordinate axis, the higher the fitness of the mice. Therefore, the degree of health in the three groups that received LPS stimulation was as follows: DHQ-H group>DHQ-L group>C+ group.

On the time dimension, the points in group C were not discrete, illustrating that the time factor had no influence on the outcome in this group. However, there was an obvious separation according to time in the three LPS-stimulated groups, which indicated that the time factor had an effect on the fitness of the mice. Among them, at 6 h, 12 h, and 24 h, the points were obviously shifted to the right side of the coordinate axis over time, and then shifted to the left side at 48 h. Combined with Figure 9(a), this illustrated that in each LPS-stimulated group, the inflammatory state of mice might be the most serious at 24 h, while at 48 h this was alleviated.

## 4. Discussion

The inflammatory response plays an important role in host defense response to pathogen invasion, tissue damage, or other environmental attacks, with the aim of restoring a state of balance [31]. Moderate inflammatory reactions can prevent the invasion of foreign pathogens and regulate the metabolism of the organism. However, excessive inflammatory reactions can lead to serious organ damage, immune dysfunction, metabolic dysregulation, and so on, which may trigger septic shock and even death [1].

DHQ is a flavonoid extracted from natural plants, and its excellent anti-inflammatory and antioxidant effects have been successively reported in the past [32–34]. However, the preventive effect of DHQ and its effect on nutrient utilization in the acute phase have not been fully reported. In the present study, we pretreated mice with 50 and 200 mg/kg BW of DHQ and subsequently established a mouse acute inflammatory response model with LPS and observed them continuously for 48 h, combined with indirect calorimetry as well as principal component analysis. We found that 2.5 mg/kg BW of LPS can induce an inflammatory response in mice. We also found that all doses of DHQ pretreatment can reduce mortality, enhance growth, potentiate immunization, enhance antioxidant status, and relieve disorders of nutrient metabolism in mice. To our knowledge, the present study was the first attempt to investigate the effects of DHQ on growth, immunity, antioxidants, and nutrient utilization in an inflammatory model in combination with indirect calorimetry, and after 48 h of continuous observation, combined with principal component analysis, to explore the dynamic changes in and protective effects of DHQ pretreatment on the inflammatory response process, from burst to resolution.

We found that in an LPS-induced mice inflammation model, pretreatment with DHQ could cause a dose-dependent reduction in mortality and that 200 mg/kg body weight DHQ pretreatment significantly increased daily food intake and daily weight gain. Our study provided evidence of DHQ alleviating anorexic and life threats in the acute phase. LPS promotes the inflammatory response by activating macrophages to produce a large number of inflammatory cytokines, which can activate neutrophils and macrophages, enhance vascular endothelial cell permeability and participate in the immune response [35]. IL-6, IL-1, and TNF- *α*, as classical inflammatory markers, were used to judge the intensity of the inflammatory response and the extent of tissue damage. The anti-inflammatory effects of DHQ have been demonstrated in previous research. Lei et al. have shown that pretreatment with DHQ (5 mg/kg, i.p) could significantly reduce the contents of TNF-*α* and IL-6 in an LPS model, alleviating the inflammatory response [36]. Similarly, in the present study, the above inflammatory cytokines were increased significantly after LPS stimulation. However, in the high-dose DHQ pretreatment group, the levels of inflammatory cytokines in the serum of the inflammatory model were inhibited, which indicated that oral administration of DHQ also has an alleviating effect on LPS-induced inflammation.

Under inflammatory conditions, in addition to secreting cytokines, macrophages and neutrophils also produce ROS radicals [37], and the presence of excessive ROS can trigger oxidative stress in organisms, especially in the liver [38]. Previous studies have pointed out that lipid peroxidation products MDA and antioxidant enzymes SOD and GSH were used as markers to evaluate oxidative stress [39]. Being stimulated by LPS could lead to a significant decrease in the levels of antioxidant enzymes (GSH-Px and T-SOD) and a significant increase in MDA content in vivo [40, 41]. In this study, similar results were also obtained in hepatic oxidative stress indicators after modeling with LPS. As an effective antioxidant [42], most of the antioxidant activity of DHQ had been confirmed in vitro or in therapy models [43, 44]. Previous reports have indicated that the antioxidant effect of DHQ may act through binding of metal ions [43] and inhibiting enzymatic reactions [45], leading to free radical formation as well as inhibiting lipid peroxidation [32]. In addition, Unver et al. [46] used an animal experiment to show that oral administration of DHQ (50 mg/kg) significantly alleviates oxidative stress damage in a cisplatin-induced lung injury model in mice. In this study, we found that DHQ pretreatment decreased liver MDA content and increased the GSH-Px and SOD contents in a dose-dependent manner in an inflammation mouse model. This indicates that DHQ could inhibit the development of oxidative damage in mice.

The stimulation of the systemic inflammatory response by LPS could change energy consumption and the metabolic pathway of nutrients in the body [47]. Serum and tissue biochemical indicators reflect the health status and metabolic function of the body [48].

In our study, Glu was slightly increased in the LPS group at 6 h, followed by a sustained decrease. Liver glycogen continued to decrease within 48 h, and LDH, a key enzyme of glycolysis, was significantly increased. Our study was similar to that of Filkins and Buchanan [49], who showed that after LPS injection in normally fed mice, blood glucose rose transiently and then decreased. This was due to a large amount of glucose being used for energy supply and repair of injury in the early phase of acute inflammation, the uptake and demand of glucose from the blood by peripheral tissues being enhanced, [50] and a large amount of liver glycogen decomposition and gluconeogenesis also being increased [51], leading to the elevation of blood glucose over a short time. Then, with the peripheral tissues exhibiting a greater demand for blood glucose than there is a supply [52], the liver glycogen depletion and serum Glu decreased. Meanwhile, endotoxins also could induce microcirculation dysfunction in the body [53], and under conditions of cellular and tissue ischemia and hypoxia, anaerobic metabolism dominated, mitochondrial oxidative phosphorylation led to a dramatic decrease in ATP production [54], and the intracellular glycolysis energy supply mechanism was activated to maintain the energy supply, becoming one of the main sources of ATP [3, 54]. Glycolytic metabolism was enhanced under conditions of low oxygen and high energy demand; thus, LDH increased. In our study, the group that underwent DHQ pretreatment, especially high-dose DHQ, experiences significantly alleviated disorders of indexes related to glucose metabolism.

In terms of lipid metabolism, both cholesterol and triglycerides derived from food or produced in the body were eventually transported into the blood, so serum TC and TG could intuitively reflect the lipid metabolism in the organism. In this study, compared with the control group, both serum TG and TC of mice in each group after LPS treatment were increased significantly, with an overall initial increase followed by a decrease within 48 h and peaking at 24 h. Meanwhile, the TG levels in the liver were also significantly increased. This trend in lipid metabolism was consistent with previous reports [55–57]. The results were mainly due to negative feedback enhancing fat mobilization at low levels of hepatic glycogen, and nonesterified fatty acids released from adipose tissue maintain metabolic energy supply [58]. It has also been reported that after LPS stimulation, hepatic fatty acid synthase transcriptional activity, and fatty acid synthesis were increased, and ketone products were decreased in the liver [59]. Meanwhile, the oxidative metabolism of fatty acids was also attenuated, especially medium- and short-chain fatty acids [60]. LPS also could decrease lipoprotein breakdown and increase blood and intrahepatic TG levels leading to hypertriglyceridemia [61, 62]. Combined with the previous report, the reasons for the elevation of TC may be large amounts of very-low-density lipoprotein and low-density lipoprotein being accumulated in the plasma, while the concentration of high-density lipoprotein was decreased and lipoprotein lipase activity decreased. These lipoproteins in the bloodstream enhanced hepatic lipid synthesis or/and decreased the clearance rate of lipids [63]. In addition, inflammatory cytokines also affect lipid metabolism, as TNF can significantly reduce the levels of key enzymes in fatty acid synthesis, can induce lipolysis [61], and can promote the accumulation of liver TG [64]. Among the IL family, IL-6 contributes to lipolysis and free fatty acid uptake in tissues [65], while IL-1 can play a role in lipid metabolism by downregulating insulin levels and lipase activity [66]. This was consistent with our results. Hawthorn leaf flavonoid extract significantly reduced serum TG and TC levels in a high-fat diet mouse model [67], and furthermore, quercetin significantly reduces serum TG and LDL levels in rats fed with a high-fat diet [68]. Gao et al. showed that [69] DHQ can regulate blood glucose homeostasis and reduce blood pressure and dyslipidemia in a rat model of metabolic syndrome. In this study, DHQ pretreatment groups had reduced contents of sera TG, TC, and TG in the liver, and high-dose DHQ could reduce liver weight (data not shown). This indicates that DHQ reduced liver lipid deposition and hyperlipidemia caused by LPS.

Serum total protein and urea nitrogen reflect the metabolism of protein in the body to a certain degree. In the present study, after LPS injection, a decrease in serum urea nitrogen was an indication of decreased efficiency in the use of dietary nitrogen [70], and a decrease in the total protein in serum indicated decreased protein synthesis. In the case of insufficient glucose supply, the protein was used as an energy source in addition to fat, protein synthesis in the body was inhibited, and a large amount of protein underwent catabolism. Meanwhile, the decrease in serum TP level in the acute phase may also be due to the increase in capillary permeability, in which a large of amount albumin enters the damaged tissue to participate in metabolism, with a consequent decrease in albumin in the blood [71]. In addition, it also has been reported that TNF- *α* can promote myofibrillar protein degradation in rats [72]. In the present study, all the DHQ pretreatment groups were seen to have experienced a regulatory effect regarding LPS-induced disorders of protein metabolism in the serum.

There was a close relationship between the health status of organisms and energy consumption. In the acute phase, inflammation leads to disorders in the metabolism of carbohydrates, fat, and protein, which intuitively manifested in the alteration of CO_2_ exhalation and O_2_ consumption, as well as nitrogen emission. Therefore, in the present trial, the metabolism and utilization of energy substances were detected by indirect calorimetry, a noninterventional method, to reflect the protective effect of DHQ in mice in the acute phase.

In the present study, we administrated LPS to mice, and the levels of both CO_2_ and O_2_ decreased significantly, then gradually increased after 18 h, in which the original circadian rhythm was broken. The decrease in CO_2_ production may be due to the anorexia of mice caused by LPS stimulation, which reduces the intake and energy supply from energy substances. Inflammation leads to abnormal distribution of systemic blood flow, hypoxia in organs or local tissues, and destroyed regulation ability of microcirculation and mitochondrial function. Therefore, oxygen consumption was reduced [73–75]. These results were largely consistent with the findings of Silverman et al. [76] and Irahara et al. [77], who administered 1 mg/kg and 5 mg/kg LPS to mice, respectively. They point out that CO_2_ and O_2_ levels were associated with the degree of inflammation. In our study, the levels of O_2_ and CO_2_ were increased in the DHQ pretreatment groups, and the high-dose DHQ group trended more towards the baseline in 48 h.

RQ can be used in indirect calorimetry to determine the relative involvement of carbohydrates, lipids, and proteins in energy production [78, 79]. The results of the RQ in our study suggest that the energy supply from carbohydrate oxidation was decreased and the dependence of energy metabolism on fat was increased under an inflammatory state. Additionally, the carbohydrate supply resumed gradually with time. However, in the DHQ-pretreated group, the RQ values were dose dependently increased, indicating that the dependency on fat supply was alleviated.

TEE reflects the total energy expenditure over a period of time, which also correlated with physiological habits and frequent night feed activity. Administration of LPS resulted in a significant decrease in TEE, which may be related to the impaired activity and feed intake of mice induced by LPS [76]. However, there was an increase in TEE in DHQ-pretreated mice, and by observation, active behaviors were more frequent in the DHQ high-dose group compared to the C+ group. The changes in TEE and RQ were detected by indirect calorimetry to assess the health status and energy needs [80] of patients in clinical medicine, coupled with internal and external nutrition, in order to give appropriate nutrition support to the patient [81]. However, there were no standardized rules of the values and changes under different disease conditions [76, 82–84]. Therefore, it was possible to evaluate the health status of the body using RQ and TEE values or change degree, but these also need to be combined with other indicators to make a comprehensive judgment.

Subsequently, we used indirect calorimetry combined with a urinary nitrogen excretion test to calculate the oxidation energy supply and proportion of three nutrient substrates, respectively. It was found that after LPS stimulation, with the enhancement of catabolism and the increase in energy material demand, the proportion of carbohydrate oxidation energy supply and carbohydrate oxidation energy supply in the total production capacity decreased significantly, and the proportion of fat and protein oxidation energy supply in the total production capacity increased significantly. Combined with the analysis of blood indicators, it was indicated that during the inflammatory phase, the energy substrate supply relationship shifted from glucose-metabolism-dominated to lipid-metabolism-dominated, and glycolysis was enhanced, oxidative phosphorylation level was weakened, glucose oxidation was limited [85], and protein catabolism was also increased. In other words, lipids and a small portion of proteins became the main energy source, which was consistent with previous studies [77]. However, the DHQ high-dose pretreatment group had increased carbohydrate oxidation energy supply and the ratio of this to the total energy supply. Although the fat oxidation energy supply was increased, the proportion of fat oxidation energy supply in the total energy as a whole decreased, as did the protein oxidation energy supply ratio. Further, the negative nitrogen balance in the body was alleviated, and the overall metabolic status was closer to that of the control group. Thus, high-dose DHQ could regulate the energy metabolism disorder of mice caused by LPS. Previous studies have reported that the continuous process of inflammation is related to nutrition and metabolism, and the proinflammatory phase initiated in acute inflammation depends on glycolysis to meet the rapid demands for high energy [86]. In the subsequent adaptive phase, which relies on fat oxidation as a fuel, fat oxidation enhancement promotes the organism to regain balance [87]; ultimately, the inflammatory state gradually tends to subside [88].

Then, through the analysis of the dynamic changes in the three kinds of energy supply nutrients, combined with PCA, it was speculated that, within the same LPS-stimulated group, the inflammatory status gradually aggravated over time, the inflammatory process tended to recover until about 24 h, and although the increase in fat oxidation supply was not observed at 48 h, the trend of fat oxidation energy supply gradually levelled off with time, in contrast to before. However, due to the complexity of multiple factors when inflammation bursts in the body, it was difficult to clearly define the stage. Our results have similarities with Bankey and Irahara's study [82] study, where they found a significant decrease in carbohydrate oxidation and fat oxidation and a significant increase in protein oxidation with increasing severity of inflammation in an LPS-stimulated mouse model. Therefore, we found that, in contrast to the C+ group, energy supply from carbohydrate oxidation and fat were both increased in the DHQ-pretreated groups as a whole from 6 h onwards, indicating that early administration of DHQ could slow down inflammation and play a protective role in mice.

After comprehensive analysis of each indicator, it could be found that carbohydrate, fat, and protein metabolism played an important role in the inflammatory process in an LPS-stimulated mouse model. It was also confirmed that the changing trend of energy supply from carbohydrate and fat oxidation could reflect the inflammatory status. However, pretreatment with DHQ was able to modulate energy metabolism disorder in mice and reduce their inflammatory state.

In conclusion, we showed that DHQ pretreatment during the acute phase improved the survival rate, immunity, antioxidant capacity, and nutrient substance metabolism disorder in mice with LPS-induced inflammation. In addition, this protective effect has been shown from the early stage of an inflammation outbreak. Taken together, our study demonstrates the potential value of DHQ as an immunopotentiator. We expect our findings to have applications in the clinical setting.

## Figures and Tables

**Figure 1:** Structure of dihydroquercetin.

**Figure 2:** DHQ improved survival and growth performance in LPS-induced mice. (a) Survival rate. (b) Average daily gain. (c) Average daily food intake. Data are expressed as the mean ± SD. Values with different superscripts are significantly difference (lower case letter: *p* < 0.05; capital letter *p* < 0.001) as determined by Tukey's test.

**Figure 3:** DHQ regulate serum and liver metabolism of nutrients parameters in LPS-induced mice. (a) Serum GLU. (b) Serum LDH. (c) Serum TG. (d) Serum TC. (e) Serum BUN. (f) Serum TP. (g) Liver glycogen. (h) Liver TG. Data are expressed as the mean ± SD. Values with different superscripts are significantly difference (lower case letter: *p* < 0.05; capital letter: *p* < 0.01) as determined by Tukey's test.

**Figure 4:** DHQ enhances liver antioxidant capacity in LPS-induced mice. (a) Liver MDA. (b) Liver SOD. (c) Liver GSH-PX. Data are expressed as the mean ± SD. Values with different superscripts are significantly difference (lower case letter: *p* < 0.05; capital letter: *p* < 0.01) as determined by Tukey's test.

**Figure 5:** DHQ reduce serum inflammatory cytokines levels in LPS-induced mice. (a) Serum TNF-*α*. (b) Serum IL-1*β*. (c) Serum IL-6. Data are expressed as the mean ± SD. Values with different superscripts are significantly difference (lower case letter: *p* < 0.05; capital letter: *p* < 0.01) as determined by Tukey's test.

**Figure 6:** DHQ pretreatment exhibit altered metabolism in LPS-challenged mice. (a) O_2_ consumption. (b) CO_2_ production (c) RQ. (d) TEE. Data are expressed as the mean ± SD. ^∗∗^*p* < 0.01 vs. the LPS group. ^#^*p* < 0.05, ^##^*p* < 0.01 vs. the LPS+DHQ group in Tukey's test.

**Figure 7:** DHQ pretreatment exhibit altered substrate utilization in LPS-challenged mice. (a) OXCHO. (b) OXCHO/TEE. (c) OXF. (d) OXF/TEE. (e) OXP. (f) OXP/TEE. Data are expressed as the mean ± SD. Values with different superscripts are significantly difference (lower case letter: *p* < 0.05; capital letter: *p* < 0.01) as determined by Tukey's test.

**Figure 8:** Correlation analysis between various indicators. Blue indicates positive correlation and red indicates negative correlation. ^∗∗^*p* < 0.01, ^∗^*p* < 0.05.

**Figure 9:** Principal component analysis (PCA). (a) Loading plot. (b) Score plots. Principal components were calculated considering all the parameters evaluated in this study. Samples were labelled according to the different treatment groups (orange: C; green: C+; violet: DHQ-L; and blue: DHQ-H) and time (+: 6 h; ●: 12 h; ▲: 24 h; ■: 48 h).

## Data Availability

The data used to support the findings of this study are included within the article.
